RETRACTED

# Clinical Efficacy of Integrated Traditional Chinese and Western Medicine in the Treatment of Eczema: A Meta-Analysis

**DOI:** 10.1155/2022/7202626

**Published:** 2022-03-03

**Authors:** Xingxing Wang, Jian Meng, Qing Wu, Jingjing Feng, Huiling Jing

**Affiliations:** ^1^Department of Dermatology, Xi'an Hospital of Traditional Chinese Medicine, Xi'an, Shaanxi 710021, China; ^2^Department of Second Surgery, Gushi County Hospital of Traditional Chinese Medicine, Xinyang, Henan 465200, China

## Abstract

**Background:**

Both traditional Chinese medicine (TCM) and Western medicine are widely applied in the treatment of eczema, but there are few reports on integrated TCM and Western medicine for eczema.

**Objective:**

This meta-analysis carried out the evaluation on the efficacy of integrated TCM and Western medicine in the treatment of eczema.

**Methods:**

PubMed, Web of Science, Embase, CNKI, and Wanfang databases were searched for all possible randomized controlled trials from 2000 to 2021. A meta-analysis of the included studies was also performed using Stata16 software.

**Results:**

A total of 16 studies including 1946 patients were included. Compared with the control group, the pooled results of the 16 studies showed that effective rate in the treatment group was higher (OR = 4.50, 95% CI: 3.16-6.40, *P* < 0.05), and the pooled data of 15 studies revealed that the cure rate was increased in the treatment group (OR = 2.60, 95% CI: 2.13-3.18, *P* < 0.05). Additionally, compared with the control group, pooled data of 11 studies demonstrated that lesion area after treatment was reduced in the treatment group (SMD = −1.91; 95% CI: -2.51, -1.31; *P* < 0.05), and pooled data of 9 studies showed that the degree of pruritus after treatment in the treatment group was lower (SMD = −1.69; 95% CI: -2.07, -1.30; *P* < 0.05).

**Conclusion:**

In comparison with Western medicine alone, integrated TCM and Western medicine are a more effective treatment for eczema, which can not only significantly improve the effective rate and cure rate but also reduce the lesion area and degree of pruritus.

## 1. Introduction

Eczema is a common chronic cutaneous inflammatory disease in clinical practice. In developed countries, 30% of children and 10% of adults are affected by this disease, while 7.5% of adults in China are affected [1]. Eczema is clinically characterized by skin redness and other changes in the skin surface, such as scaling, swelling, hair follicle protrusion, and chronic scratching-caused skin thickening, often accompanied by intense pruritus [2]. Eczema can appear on the skin of the whole body, with different predilection sites at different ages. The disease is long-lasting, causing great disruption to the work and life of patients and increasing the financial burden on patients and their caregivers [3].

RETRACTED

The exact pathophysiological mechanism of eczema has not been fully elucidated, and there is no optimal cure [4]. Western medicine usually uses glucocorticoids, antibacterial drugs, H1 receptor antagonists, immunomodulators, and other drugs to treat eczema [5]. However, high recurrence rates, side effects, and drug resistance are a constant concern [6]. Therefore, it is necessary to develop therapeutically effective agents with few side effects. Traditional Chinese medicine (TCM) has classical prescriptions, empirical prescriptions, Chinese patent medicines, and external treatments [7]. For example, Xiao-Feng-San has been shown to be effective in eczema [8]. Tripterygium wilfordii Hook F is also listed as an adjuvant drug for eczema treatment [9]. However, some herbs exhibit serious intrinsic liver, kidney, and gastrointestinal toxic reactions with regular clinical use [10]. Therefore, considering the efficacy and safety, some studies have combined TCM and Western medicine to treat eczema in recent years and have shown significant clinical efficacy and safety [11–13]. However, the sample size included in each study is small, and there is a lack of systematic assessment of the efficacy and safety of combining Chinese and Western medicine in the treatment of eczema. In this study, we systematically evaluated the clinical efficacy of integration of traditional and Western medicine in the treatment of eczema by conducting a meta-analysis of randomized controlled trials, with the aim of providing a clinical basis for treatment.

## 2. Materials and Methods

### 2.1. Retrieval Methods

PubMed, Web of Science, Embase, CNKI, and Wanfang databases were searched for all possible randomized controlled trials from 2000 to 2021, without limitations on language and publication status (published, unpublished, and ongoing). The keywords were as follows: (“integrated traditional Chinese and Western medicine”) and (“eczema”) and (“clinical effect”).

### 2.2. Inclusion and Exclusion Criteria

The inclusion criteria were as follows: (1) study type: randomized controlled trials with or without blind method; (2) study subjects: adult patients diagnosed with eczema according to the diagnostic criteria of Western medicine for clinical dermatology or eczema diagnosed according to the criteria of TCM differentiation, informed consent obtained from patients, patients without administration of any other type of drugs, patients without other underlying diseases or mental illness, and patients with good compliance; (3) intervention: the treatment group was given integrated TCM and Western medicine, while the control group was treated with conventional Western medicine alone; and (4) outcome measures: effective rate, cure rate, lesion area after treatment [14], and degree of pruritus after treatment.

RETRACTED

The exclusion criteria were as follows: (1) duplicate article; (2) duplicate data; (3) incomplete or unavailable data; and (4) reviews, conference abstracts, and case reports.

### 2.3. Data Extraction

Based on the screening criteria mentioned above, two authors independently screened studies by reading titles and abstracts. Then, the full text of potential included studies was retrieved for further assessment. During this process, the disagreement was resolved through the discussion within the research group. The following data were extracted: basic characteristics of participants, intervention measures, and outcome measures.

### 2.4. Statistical Analysis

Stata16.0 software was a statistical tool utilized for data analysis. Dichotomous data were presented as odds ratios (OR) with 95% confidence intervals (CI), while continuous data are presented as standardized mean difference (SMD) with 95% CI. In case of heterogeneity (*P* > 0.05, *I*^2^ < 50%), the fixed-effects model was employed for analysis; Otherwise, the random-effects model was adopted. Publication bias was assessed by funnel plots and Begg's and Egger's tests. Sensitivity analysis was also performed to determine the stability of meta-analysis results.

## 3. Results

### 3.1. Retrieval Results

Initially, 161 articles were retrieved, and then, 68 articles were included after excluding duplicate literature. Next, 26 articles were excluded after reading titles and abstracts. Ultimately, 16 studies [11–13, 15–27] were included after reading the full text. The literature screening process is shown in Figure 1.

### 3.2. Characteristics of Included Studies

The 16 studies included 1946 subjects, 1034 in the treatment group, and 912 in the control group. They were all randomized controlled clinical studies, with sample sizes ranging from 58 to 365 and study time from 10 months to 2 years. The age of the study subjects varied from 1 to 65 years, with a gender ratio of 1.30 (1101 : 845). Basic characteristics of the included studies are shown in Table 1.

### 3.3. Meta-Analysis Results

#### 3.3.1. Effective Rate and Cure Rate after Treatment

The heterogeneity of 16 literatures [11–13, 15–27] on the effective rate was tested, and the fixed-effects model was finally utilized (*I*^2^ = 0.00%, *P* = 0.974). Meta-analysis results suggested a significant difference in the effective rate, which was higher in the treatment group than that in the control group (OR = 4.50, 95% CI: 3.16-6.40, *P* < 0.05) (Figure 2(a)).

RETRACTED

The heterogeneity of 15 literatures [11–13, 15, 16, 18–27] on the cure rate was tested, and the fixed-effects model was finally utilized (*I*^2^ = 0.00%, *P* = 0.957). Pooled result suggested a significant difference in the cure rate, which was higher in the treatment group than that in the control group (OR = 2.60, 95% CI: 2.13-3.18, *P* < 0.05) (Figure 2(b)).

#### 3.3.2. Lesion Area and Degree of Pruritus after Treatment

The heterogeneity of 11 literatures [11–13, 15, 16, 18, 19, 21–23, 25] on the lesion area after treatment was tested, and the random-effects model was finally utilized (*I*^2^ = 95.8%, *P* < 0.05). Pooled result suggested a significant difference in the lesion area after treatment, which was reduced in the treatment group compared with the control group (SMD = −1.91; 95% CI: -2.51, -1.31; *P* < 0.05) (Figure 2(c)).

The heterogeneity of 9 literatures [11–13, 15, 16, 21–24] on the degree of pruritus after treatment was tested, and the random-effects model was finally utilized (*I*^2^ = 85.1%, *P* < 0.05). Meta-analysis results showed that the degree of pruritus after treatment in the treatment group was significantly improved compared with the control group (SMD = −1.69, 95% CI: -2.07, -1.30; *P* < 0.05) (Figure 2(d)).

### 3.4. Publication Bias

#### 3.4.1. Effective Rate and Cure Rate

The Egger test (*t* = 2.55, *P* = 0.023) and Begg's test (*Z* = 0.41, *P* = 0.685) of the effective rate indicated no publication bias in this included literature. Similarly, Egger test (*t* = 4.60, *P* < 0.05) and Begg's test (*Z* = 0.69, *P* = 0.488) of the cure rate also showed no publication bias. Further, the inverted funnel plots were plotted with the effective rate and cure rate as indicators, respectively, showing that the scatter distribution was basically symmetrical and thus suggesting little possibility of publication bias in this analysis (Figures 3(a) and 3(b)).

#### 3.4.2. Lesion Area and Degree of Pruritus after Treatment

The Egger test (*t* = 0.30, *P* = 0.773) and Begg's test (*Z* = 1.71, *P* = 0.087) of the lesion area indicated the possibility publication bias in this included literature. Similarly, Egger's test (*t* = −0.21, *P* = 0.836) and Begg's test (*Z* = 1.36, *P* = 0.175) of the degree of pruritus showed no significant publication bias. Further, the inverted funnel plots were plotted with effective rate and cure rate as indicators, respectively, showing that the scatter distribution was basically symmetrical and thus suggesting little possibility of publication bias in this analysis (Figures 3(c) and 3(d)).

### 3.5. Sensitivity Analysis

Sensitivity analysis was performed for all four indicators, and the results were as follows: effective rate (OR: 4.50; 95% CI: 3.16, 6.40), cure rate (OR: 2.60; 95% CI: 2.13, 3.18) (Figures 4(a)–4(b)), lesion area (SMD: -1.91; 95% CI: -2.51, -1.31), and degree of pruritus (SMD: -1.69; 95% CI: -2.07, -1.30) (Figures 4(c) and 4(d)). Compared with the original results, the statistical significance did not change, and the scatters of each study were within the CI, suggesting robust meta-analysis results.

RETRACTED

## 4. Discussion

Eczema, clinically, is a skin inflammation with a high incidence that occurs in different age groups, especially infants and children. This is a disease that has a profound impact on the social, emotional, and physical health of patients, as well as economic status [28].

The treatment of eczema is mainly based on conventional Western medicine, such as prednisone, prednisolone, and triamcinolone acetonide, which is applied for short-term control of significant erythema of eczema, but not for long-term treatment [29]. Because Western medicine causes some side effects in the treatment of eczema, specifically, corticosteroids have many side effects, including increased risk of infection, hypertension, impaired glucose tolerance, weight gain, gastritis, decreased bone mineral density, adrenal suppression, ophthalmic complications (including cataracts and glaucoma), sleep disorders, and emotional lability [30]. Cyclosporine A (cyclosporine) can lead to adverse effects including increased risk of infections, renal toxicity, hypertension, hirsutism, gingival hyperplasia, tremor, and skin malignancies and lymphomas [31, 32]. Methotrexate has the following potential side effects: nausea and gastrointestinal upset (usually avoided by subcutaneous injection), oral and mucosal ulceration, myelosuppression, increased risk of infection, hepatotoxicity, and pulmonary fibrosis [33, 34]. Mycophenolate mofetil also usually causes gastrointestinal upset [35]. Collectively, Western medicine can significantly improve the clinical symptoms of eczema, but their side effects are many and more serious, especially for long-term treatment. TCM is also effective in the treatment of eczema. Some studies have shown that patients with urticaria who take triptolide are more likely to develop gastrointestinal reactions and reproductive damage and can also lead to abnormal liver function [6, 36]. Therefore, investigators have begun to use measures such as dosing and using low doses of drugs to reduce toxic effects. Liu et al. [37] confirmed that Tripterygium wilfordii combined with topical glucocorticoids had a significant effect on eczema. Therefore, many patients with eczema can choose Chinese herbal medicine as a complementary medicine to Western medicine to treat eczema.

RETRACTED

In this meta-analysis, the differences in clinical efficacy were compared between integrated TCM and Western medicine and Western medicine alone in the treatment of eczema, thus providing theoretical guidance for subsequent clinical practice. The results showed that the effective rate of the former was higher than that of the latter, and so was the cure rate. Additionally, compared with the control group, lesion area after treatment in the treatment group was reduced, and the degree of pruritus in the treatment group was improved. Taken together, integrated TCM and Western medicine are effective for eczema, which can not only significantly improve the effective rate and cure rate but also reduce the lesion area and degree of pruritus.

Our study still has some limitations. First, there is some heterogeneity of the included trials, which may lead to overestimation or underestimation of the differences between the groups. Second, the incidence of eczema varies greatly among age groups, which was most common in children, but no adjustment for age was made in this meta-analysis. Third, type of drugs and administration methods are various, but there are no specific drugs, administration methods, doses, and frequencies mentioned in the study, which potentially lead to some bias.

In summary, compared with Western medicine alone, integrated TCM and Western medicine are an effective therapy for eczema, which can not only significantly improve the effective rate and cure rate but also reduce the lesion area and degree of pruritus. Integrated TCM and Western medicine can significantly relieve the clinical symptoms, deserving clinical application.

## Figures and Tables

**Figure 1:** Literature screening process.

**Figure 2:** Forest plots of the effective rate (a), cure rate (b), lesion area (c), and degree of pruritus (d).

**Figure 3:** Funnel plots of the lesion area (a), degree of pruritus (b), effective rate (c) and cure rate (d).

**Figure 4:** Sensitivity analysis of the effective rate (a), cure rate (b), lesion area (c), and degree of pruritus degree (d).

**Table 1:** The basic characteristics of inclusion in the literature.

Study	Year	Sample time (year.month)	Cases (treatment/control)	Age (years)		Gender (male/female)		Study design	Outcome measures
				Treatment group	Control group	Treatment group	Control group		
Qiu Changan	2018	2017.02-2018.02	57/57	35.08 ± 7.25	34.85 ± 7.34	28/29	24/33	RCT	①+②+③+④
Tang Changren	2015	2011.01-2013.12	42/42	42.3 ± 8.7	43.9 ± 9.5	26/18	24/19	RCT	①+②+③+④
Peng Leilei	2016	2012.04-2014.04	90/90	20-70	18-66	47/43	50/40	RCT	①+②+③+④
Wen Yunbo	2016	2013.07-2014.07	40/40	40.3 ± 3.5	43.5 ± 4.7	21/19	24/16	RCT	①+②+③+④
Huang Xiang	2019	2016.05-2018.05	62/62	44.73 ± 3.85	46.28 ± 3.75	32/30	34/28	RCT	①+②+③+④
Ma Hui	2016	2014.02-2015.02	45/45	38.00 ± 2.58	39.00 ± 3.87	22/23	22/23	RCT	①
Miu Shidong	2014	2011.03-2013.03	218/147	27.96 ± 3.25	28.00 ± 3.19	133/85	87/60	RCT	①+②+③
Cai Xinjie	2014	2007.10-2013.10	80/40	18-65	18-65	54/26	24/16	RCT	①+②+③
Li Ting	2015	2011.03-2013.10	45/44	30.95 ± 10.19	28.34 ± 12.65	26/19	29/16	RCT	①+②
Tang Zhongfen	2016	2014.10-2015.10	50/50	41.6 ± 13.4	40.9 ± 7.8	32/18	27/23	RCT	①+②+③+④
Zhang Cunxue	2015	2012.06-2014.06	91/82	1.13 ± 0.87	1.34 ± 0.69	51/40	45/37	RCT	①+②+③+④
Kong Danyang	2019	2017.08-2018.06	40/40	63.8 ± 7.2	60.7 ± 5.4	23/17	22/18	RCT	①+②+③+④
Yang Hui	2018	2016.01-2017.01	29/29	36.7 ± 4.8	36.8 ± 4.6	17/12	16/13	RCT	①+②+④
Ye Zhaowei	2017	2015.09-2016.09	35/34	20 ± 1.87	19 ± 1.69	19/16	20/14	RCT	①+②+③
Luo Lina	2018	2015.02-2017.02	60/60	40.12 ± 4.03	40.26 ± 4.06	36/24	38/22	RCT	①+②
Gong Chaochao	2019	2017.09-2018.12	50/50	23-65	23-65	27/23	21/29	RCT	①+②

Note: RCT: randomized controlled trial; NR: not reported; ①: total effective rate; ②: cure rate; ③: lesion area after treatment; ④: degrees of pruritus after treatment.

RETRACTED

## Data Availability

The data that support the findings of this study are available from the corresponding author upon reasonable request.
